RETRACTED

# Targeting and Therapy of Glioblastoma in a Mouse Model Using Exosomes Derived From Natural Killer Cells

**DOI:** 10.3389/fimmu.2018.00824

**Published:** 2018-04-23

**Authors:** Liya Zhu, Ji Min Oh, Prakash Gangadaran, Senthilkumar Kalimuthu, Se Hwan Baek, Shin Young Jeong, Sang-Woo Lee, Jaetae Lee, Byeong-Cheol Ahn

**Affiliations:** Department of Nuclear Medicine, School of Medicine, Kyungpook National University, Kyungpook National University Hospital, Daegu, South Korea

**Keywords:** exosomes, natural killer cells, tumor targeting, immunotherapy, glioblastoma

## Abstract

**Objective:**

Glioblastoma is a highly aggressive primary brain tumor that is resistant to radiotherapy and chemotherapy. Natural killer (NK) cells have been used to treat incurable cancers. Recent studies have investigated the effectiveness of NK-cell-derived exosomes (NK-Exo) for treating incurable cancers such as melanoma, leukemia, and neuroblastoma; however, NK-Exo have not been used to treat glioblastoma. In the present study, we investigated the antitumor effects of NK-Exo against aggressive glioblastoma both *in vitro* and *in vivo* and determined the tumor-targeting ability of NK-Exo by performing fluorescence imaging.

**Methods:**

U87/MG cells were transfected with the enhanced firefly luciferase (effluc) and thy1.1 genes; thy1.1-positive cells were selected using microbeads. U87/MG/F cells were assessed by reverse transcription polymerase chain reaction (RT-PCR), western blotting, and luciferase-activity assays. NK-Exo were isolated by ultracentrifugation, purified by density gradient centrifugation, and characterized by transmission electron microscopy, dynamic light scattering (DLS), nanoparticle-tracking analysis (NTA), and western blotting. Cytokine levels in NK-Exo were compared to those in NK cells and NK-cell medium by performing an enzyme-linked immunosorbent assay (ELISA). NK-Exo-induced apoptosis of cancer cells was confirmed by flow cytometry and western blotting. *In vivo* therapeutic effects and specificity of NK-Exo against glioblastoma were assessed in a xenograft mouse model by fluorescence imaging. Xenograft mice were treated with NK-Exo, which was administered seven times through the tail vein. Tumor growth was monitored by bioluminescence imaging (BLI), and tumor volume was measured by ultrasound imaging. The mice were intraperitoneally injected with dextran sulfate 2 h before NK-Exo injection to decrease the liver uptake and increase the tumor specificity of NK-Exo.

**Results:**

RT-PCR and western blotting confirmed the gene and protein expression of effluc in U87/MG/F cells, with the bioluminescence activity of U87/MG/F cells increasing with an increase in cell number. NTA and DLS results indicated that the size of NK-Exo was ~100 nm, and the western blot results confirmed that NK-Exo expressed exosome markers CD63 and Alix. We confirmed the *in vitro* cytotoxic effects of NK-Exo on U87/MG/F cells by performing BLI, and the killing effect on U87/MG and U87MG/F cells was measured by CCK-8 and MTT assays (*p* < 0.001). ELISA results indicated that NK-Exo contained tumor necrosis factor-α and granzyme B. *In vivo* NK-Exo treatment inhibited tumor growth compared to in control mice (*p* < 0.001), and pretreatment of xenograft mice with dextran sulfate 2 h before NK-Exo treatment increased the antitumor effect of NK-Exo (*p* < 0.01) compared to in control and NK-Exo-alone-treated mice.

RETRACTED

**Conclusion:**

NK-Exo targeted and exerted antitumor effects on glioblastoma cells both *in vitro* and *in vivo*, suggesting their utility in treating incurable glioblastoma.

## Introduction

Glioblastoma is a highly aggressive primary brain tumor, with ~210,000 new cases diagnosed annually worldwide (1). Outcomes for patients with glioblastoma remain poor after multimodal therapy, which includes surgical resection, radiotherapy, and chemotherapy. Moreover, the highly infiltrative nature of glioblastoma increases the rate of tumor recurrence after conventional treatment (2, 3). Immunotherapy offers a mechanistic approach that differs from conventional treatments. Moreover, immunotherapy has been successfully used to treat other cancers, indicating its potential for treating glioblastoma (4–7). Natural killer (NK) cells were discovered >40 years ago and have been found to control microbial infections and tumor progression, with >50 clinical trials assessing NK cells as of March 2017 (http://clinicaltrials.gov). NK cells mediate the cytotoxicity of target cells independently of any previous activation (5, 8–10); however, effective immunotherapy of glioblastoma is associated with several limitations, including the tightly regulated interface between the bloodstream and central nervous system, an immune-privileged site, and evasion of immune surveillance because of the blood–brain barrier (BBB) (8, 9). Exosomes have recently gained attention because of their role in onco-immunology, as they represent nanovesicles capable of encompassing several molecules and enabling delivery of their contents to target cells (10, 11).

Exosomes are nanovesicles released by nearly all cells in the body to deliver several molecules, including proteins, lipids, and nucleic acids, to target cells (12–14). Exosomes are non-viable and can be engineered to incorporate therapeutic mRNAs, short-interfering RNAs, and chemotherapeutic molecules, thus making them good candidates for cancer treatment (11, 15–17). Exosomes contain variable proteins depending on their parent cells. For example, exosomes from tumor cells contain tumor antigens, platelet-derived exosomes contain coagulation factors, and exosomes from dendritic cells express toll-like-receptor ligands (18, 19). The biological functions of exosomes also differ depending on the physiological conditions and cells from which they originate. However, exosomes share certain characteristic protein compositions, such as expression and display of CD9, CD63, and CD8, and proteins involved in endocytosis and cargo sorting, such as flotillin and tumor-susceptibility gene 101 protein (18, 20–23). The use of exosomes in cancer treatment has been explored, with a previous study showing that mesenchymal stem cell (MSC)-derived exosomes exert antitumor effects by inhibiting mitogen-activated protein (MAP) kinase pathways (24). Moreover, exosomes derived from microRNA (miR)-146b-expressing MSCs significantly reduced glioblastoma growth in a rat model of primary brain tumor (25). Exosomes derived from dendritic cells show strong immune activation and have been used to treat tumors in the preclinical stage (e.g., NCT01159288) (26, 27). Because of their size, exosomes can be exploited to carry cargo across the BBB (10, 28–30). For example, macrophage-derived exosomes loaded with catalase protect mice from oxidative stress and inhibit neurodegeneration *in vivo* (11). A previous study showed that NK cells release exosomes under both resting and activated conditions (31, 32). We previously found that NK-cell-derived exosomes express killer proteins [i.e., Fas ligand (FasL) and perforin] and inhibit cancer growth in a xenograft animal model (22). These findings demonstrate that, in contrast to other lymphocytes, NK cells secrete exosomes in a constitutive manner independently of their activation status. This suggests that NK-cell-derived exosomes exhibit effective immunological functions even in the absence of specific stimuli (32).

RETRACTED

A previous study showed that intratumoral injection of NK-cell-derived exosomes (NK-Exo) exerts excellent therapeutic effects by inhibiting cancer growth in a xenograft animal model (22). However, exosomes should be administered intravascularly and not intratumorally for treating systemic cancers. Moreover, the specificity of intravenously administered NK-Exo is critical for managing disseminated cancers. In this study, we isolated exosomes from NK-cell culture medium by ultracentrifugation and density gradient ultracentrifugation, followed by confirmation of the antitumor effect of NK-Exo and underlying mechanisms, using bioluminescence imaging (BLI), fluorescence-activated cell sorting (FACS), and western blotting. Additionally, the *in vivo* and *ex vivo* tumor specificity and immunotherapeutic effects of NK-Exo were confirmed using a xenograft mouse model of glioblastoma. We observed that the biodistribution of NK-Exo after repeated intravenous injections did not induce body weight loss or hepatic injury in the xenograft mouse model.

## Materials and Methods

### Cell Lines

The human glioblastoma cell line U87/MG and human NK cell line NK92-MI were obtained from American Type Culture Collection (ATCC, Manassas, VA, USA). U87/MG cells were cultured in RPMI 1640 medium (Hyclone, Logan, UT, USA) supplemented with 10% fetal bovine serum (Gibco, Grand Island, NY, USA) and 1% penicillin–streptomycin (Hyclone). NK92-MI cells were cultured in stem cell growth medium (CellGro, Freiburg, Germany) supplemented with 2% exosome-depleted human serum (ultracentrifuged at 100,000 × *g* for 18 h) and 1% penicillin–streptomycin, at 37°C in 5% CO_2_. U87/MG cells were transfected with a recombinant retrovirus containing a plasmid that showed enhanced expression of firefly luciferase (effluc) and thy1.1 genes, driven by a long terminal-repeat promoter (Retro–LTR–effluc–thy1.1). Thy1.1-positive cells were sorted from U87/MG cells expressing both effluc and thy1.1 genes using a magnetic cell sorter (Miltenyi Biotec, Bergisch Gladbach, Germany). Reverse transcription polymerase chain reaction (RT-PCR) and western blotting were performed to confirm the expression of effluc mRNA and protein, respectively. Established stable cells expressing both effluc and thy1.1 genes were referred to as U87/MG/F cells.

### Luciferase Activity of U87/MG/F Cells

U87/MG and U87/MG/F cells were seeded at various densities into clear-bottom black 96-well plates. After 24 h incubation, the cells were treated with 3 µL (3 mg/mL) d-luciferin, and their effluc activity was measured using a Lumina III *in vivo* imaging system (Perkin-Elmer, Waltham, MA, USA).

### Exosome Isolation

Natural killer-92MI cells were cultured in 75-cm^3^ flasks containing fresh culture medium for 3–4 days, and then, the medium was collected and used as conditioned medium. The conditioned medium was centrifuged at 1,500 × *g* for 3 min, 2,000 × *g* for 15 min, and 3,000 × *g* for 20 min at 4°C to remove the cells and debris. The supernatant was filtered through a 0.22-µm filter to remove large particles and then centrifuged at 100,000 × *g* for 1 h to obtain the NK-Exo pellet. The pellet containing NK-Exo was diluted with phosphate-buffered saline (PBS) and centrifuged at 100,000 × *g* (33). NK-Exo were purified by density gradient ultracentrifugation. The pellet obtained was resuspended in PBS, stored at −80°C, and used within 1 month. All ultracentrifugation steps were performed at 4°C in an Optima L-100 XP ultracentrifuge (Beckman Coulter, Brea, CA, USA). Protein content in NK-Exo was determined using the BCA protein assay kit (Pierce, Rockford, IL, USA).

RETRACTED

### Transmission Electron Microscopy (TEM)

Transmission electron microscopy was performed to identify the purified exosomes. Exosome pellets were suspended in 50 µL 2% paraformaldehyde, and the resultant exosome suspension was covered with Formvar-carbon-coated EM grids to promote the absorption of exosomes onto membranes over 20 min in a dry environment at room temperature. The grids were then placed directly on a drop of 1% glutaraldehyde and incubated for 5 min to remove the negative background. The grids were washed seven times with distilled water for 2 min each and examined using an HT 7700 transmission electron microscope (Hitachi, Tokyo, Japan) operated at 100 kV.

### Dynamic Light Scattering (DLS) and Nanoparticle Tracking Analysis (NTA)

Dynamic light scattering was performed using a zeta-potential and particle-size analyzer (ELSZ-2000; Otsuka Electronics Co., Ltd., Osaka, Japan). The size, distribution, and number of particles in the exosomal formulations were determined by NTA using a 0.01 mg/mL NK-Exo formulation that was prepared and evaluated using a NanoSight LM10 instrument (Malvern Instruments, Malvern, UK) equipped with NTA 3.0 analytical software (Malvern Instruments). All experiments were performed at 1:1,000 dilution, which provided particle concentrations of ~6 × 10^7^/mL. Each experiment was performed in triplicate.

### Western Blot Analysis

Natural killer-Exo were treated with radioimmunoprecipitation assay buffer and vortexed three times for 10 min each to promote lysis. The lysates were centrifuged at 13,200 × *g* for 20 min and the supernatant was collected. Proteins (50 µg) present in the supernatant were resolved by sodium dodecyl sulfate polyacrylamide gel electrophoresis, followed by transfer to polyvinylidene fluoride membranes (Millipore, Billerica, MA, USA). After blocking, the membranes were incubated overnight at 4°C with primary antibodies against CD63, Alix, GM130, calnexin, perforin, and FasL (Abcam, Cambridge, UK). The membranes were washed three times for 10 min each in washing buffer (Tris-buffered saline and Tween 20) with shaking and then incubated with secondary antibodies for 1 h at room temperature. The membranes were washed again for 10 min three times, and the bands obtained were visualized using an enhanced chemiluminescence detection kit (Amersham plc, Amersham, UK).

RETRACTED

### Cytotoxicity Assay

Natural killer-Exo cytotoxicity toward glioblastoma cells was determined by BLI using the Cell Counting Kit-8 (CCK-8; Dojindo Molecular Technologies, Tokyo, Japan) and 3-(4, 5-dimethylthiazolyl-2)-2, 5-diphenyltetrazolium bromide (MTT) assay (Generay Biotech Co., Ltd., Shanghai, China). U87/MG/F cells cultured in serum-free medium containing different concentrations (5 and 20 µg) of NK-Exo in 96-well plates for different durations (6, 12, and 24 h) were used for BLI. For the CCK-8 assay, U87/MG/F and U87/MG cells were incubated with different concentrations of NK-Exo in 96-well plates for 24 h, followed by addition of 10 µL CCK-8 solution to each well and incubation of the plates for 2 h in a humidified incubator. Absorbance was measured at 450 nm using a microplate reader. For the MTT assay, U87/MG/F and U87/MG cells were treated with NK-Exo for 24 h, and 100 µL of serum-free medium and 0.5 mg/mL MTT solution were added to each well. After 2-h incubation, the medium was removed and 100 µL dimethyl sulfoxide was added, followed by absorption measurement at 550 nm.

### Cell-Uptake Assay

Cell-uptake of NK-Exo was assessed using a modified chemical protocol (34). The NK-Exo suspension was incubated with a fluorescent lipophilic tracer [2-(5-(1, 3-dihydro-3, 3-dimethyl-1-octadecyl-2H-indol-2-ylidene]-1, 3-pentadienyl)-3, 3-dimethyl-1-octadecyl-perchlorate (DiD; Invitrogen, Carlsbad, CA, USA)]for 20 min at room temperature. NK-Exo were washed three times with PBS and centrifuged at 100,000 × *g* for 1 h. The obtained supernatant was removed, and exosomes in the pellet were resuspended in PBS. Next, 20 µg DiD-labeled NK-Exo were incubated with U87/MG/F cells for 1 and 3 h at 37°C. After incubation, chamber wells were washed five times with PBS and then cells were fixed with 4% paraformaldehyde for 20 min. The samples were covered with Vectashield mounting medium containing 4′,6-diamidino-2-phenylindole (Vector Laboratories, Burlingame, CA, USA), washed five times with PBS, and examined using a confocal laser microscope (LSM 800 with Airyscan; Zeiss, Jena, Germany).

### Quantification of Apoptosis

Natural killer-Exo cytotoxicity against glioblastoma cells was determined by performing annexin V-FITC/propidium iodide (PI) double staining with an annexin V-FITC kit (BD Biosciences, Franklin Lakes, NJ, USA) as described previously (22). U87/MG/F cells were incubated with 20 µg NK-Exo for 24 h, harvested, washed, centrifuged, and resuspended in binding buffer to achieve a concentration of 1 × 10^6^ cells/mL. After adding annexin V and PI dye, the cells were gently mixed and incubated in the dark for 15 min at room temperature. Binding buffer (400 µL) was added to each tube and flow cytometry was performed using the FACSCalibur system (BD Biosciences).

RETRACTED

Western blot analysis was performed to confirm NK-Exo-induced apoptosis of cancer cells. This was conducted by measuring the levels of apoptotic pathway marker proteins, caspase-3, cleaved caspase-3, and cleaved polyADP ribose polymerase (PARP), as well as cell-proliferation pathway proteins, phosphorylated (p)-AKT, and p-extracellular signal-regulated kinase (ERK), using specific antibodies (Cell Signaling Technology, Danvers, MA, USA). Moreover, the levels of phosphatase and tensin homolog (PTEN), a key tumor suppressor in the phosphatidylinositol-3 kinase (PI3K)/AKT pathway (35, 36), and p38, which is involved in the MAP kinase pathway (24, 37, 38), were detected in NK-Exo-treated cancer cells. Both PTEN and p38 increase the levels of reactive oxygen species and activate the caspase-3 pathway (24, 27, 38). Intensities of protein bands were visualized and analyzed using ImageLab software (v3.0; Bio-Rad, Hercules, CA, USA).

### Enzyme-Linked Immunosorbent Assay (ELISA)

Cytokines present in NK-Exo were determined by ELISA, using 1 × 10^6^ NK cells seeded in a flask containing serum-free medium for 72 h. The medium was collected into a centrifuge tube and centrifuged at 1,500 × *g* and 4°C for 10 min. NK cells and NK-Exo were then added to 0.5 mL radioimmunoprecipitation assay buffer, incubated on ice, and centrifuged at 13,000 × *g* and 4°C for 10 min. Granzyme B and tumor necrosis factor (TNF)-α levels in NK cells, NK-Exo, and NK-cell medium were determined using the respective ELISA kits (eBioscience, San Diego, CA, USA).

### Animal Experiments

*In vivo* analysis was performed using specific pathogen-free, 6-week-old, female BALB/c nude mice (Hamamatsu, Shizuoka, Japan). All animal experiments were performed in accordance with the National Institutes of Health guidelines for the care and use of laboratory animals (National Institutes of Health, Bethesda, MD, USA), and the protocols were approved by the Committee for Handling and Use of Animals of Kyungpook National University (Daegu, South Korea).

### Biodistribution and Tumor Specificity of NK-Exo in the Mouse Model

Natural killer-Exo were labeled with DiD and fluorescence lifetime imaging (FLI) of NK-Exo was performed using an *in vivo* imaging system. For this, 5 × 10^6^ U87/MG/F cells were subcutaneously injected into mice, which were randomly divided into three groups after 42 days. The mice were then intraperitoneally injected with dextran sulfate. Both untreated and mice pretreated with dextran sulfate received intravenous injections of 100 µg fresh DiD-labeled NK-Exo after 2 h and were subjected to FLI at different time points. Background autofluorescence was eliminated using imaging controls from mice that were not injected with NK-Exo. The organs and tumors of mice were harvested, *ex vivo* FLI was performed, and the images obtained were quantified using software. To confirm the ability of NK-Exo to cross the BBB and exert a therapeutic effect, an orthotopic brain-tumor model was also used, and the biodistribution of DiD-labeled NK-Exo was measured after intravenous injection. The brains from mice were also collected for this *ex vivo* study.

RETRACTED

### NK-Exo-Based Immunotherapy and Confirmation of Side Effects

The therapeutic effect of NK-Exo was determined using a tumor xenograft mouse model (*n* = 18). Briefly, mice were subcutaneously injected with 5 × 10^6^ U87/MG/F cells. After 10 days, mice were intravenously injected with 100 µg of NK-Exo suspension in PBS every 2 days for 14 days. Moreover, the mice were treated with dextran sulfate to block scavenger receptor A (SR-A) and prevent uptake of NK-Exo into the liver, as reported previously (21). Tumors were subjected to BLI every 3 days until 14 days after treatment, and ultrasound three-dimensional imaging (S-Sharp Corporation, New Taipei City, Taiwan) was performed to measure tumor volume. *Ex vivo* analysis was performed after 14 days. After sacrificing the mice, the tumors were subjected to BLI using an *in vivo* imaging system and their weights were measured. The body weight of the mice was determined every 4 days to confirm the long-term safety of NK-Exo treatment. The liver, lungs, spleen, and heart were harvested after all experiments and stained with hematoxylin and eosin to determine the side effects of *in vivo* NK-Exo treatment.

### Statistical Analysis

All quantitative data are expressed as the mean ± SD. Student’s *t-*test or one-way analysis of variance, followed by Scheffe’s *post hoc* test, was performed for normally distributed data, while Mann–Whitney *U* test was performed for non-normally distributed data, using SPSS version 22.0 (SPSS, Inc., Chicago, IL, USA). Statistical significance was determined at *p* < 0.05.

## Results

### NK-Exo Production and Characterization

Natural killer -Exo were isolated by ultracentrifugation and purified by density gradient centrifugation. NK-Exo morphology was analyzed by TEM, size was determined by NTA and DLS, and purity was determined by western blotting. We observed that NK-Exo were round with a complete membrane structure and a size of ~100 nm (Figure 1A). Their size was further characterized and confirmed by NTA and DLS (Figure 1B). Western blot analysis indicated that NK-Exo contained typical exosomal proteins (CD63 and Alix) and lacked cellular proteins (GM130 and calnexin) (Figure 1C). These results indicated that NK-Exo lacking cellular proteins were successfully isolated from NK-cell culture medium by ultracentrifugation.

RETRACTED

**Figure 1:** Verification of isolated natural killer (NK)-Exo. **(A)** Morphology of isolated NK-Exo was determined by transmission electron microscopy (scale bar, 500 and 100 nm). **(B)** Size of NK-Exo was measured by nanoparticle-tracking analysis and dynamic light scattering. **(C)** Expression of exosome markers CD63 and Alix was confirmed by western blotting.

### Reporter-Gene Expression and Activity in U87/MG/F Cells

Human glioblastoma cells were transfected with a reporter-gene system and examined by BLI, RT-PCR, and western blotting to measure reporter-gene expression. The results of BLI indicated that the luciferase signal strongly increased along with increasing cell number (*R*^2^ = 0.92) (Figures S1A,B in Supplementary Material). RT-PCR and western blotting indicated the mRNA and protein expression, respectively, of effluc in transfected U87/MG/F cells (Figures S1C,D in Supplementary Material).

### NK-Exo Cytotoxicity Against Glioblastoma Cells

Natural killer-Exo cytotoxicity against glioblastoma cells was determined by culturing U87/MG/F cells with various NK-Exo concentrations; these cells were subjected to BLI at various time points. NK-Exo cytotoxicity was determined by analyzing the reporter-gene signal in U87/MG/F cells (Figure 2). Our results showed that NK-Exo exerted cytotoxic effects toward glioblastoma cells in a time- and dose-dependent manner. Particularly, incubation of tumor cells with 20 µg NK-Exo for 24 h nearly completely eliminated BLI signals (*p* < 0.001; Figure 2C). Parent U87/MG cells were also used to confirm NK-Exo cytotoxicity by performing the CCK-8 and MTT assays. The CCK-8 results showed that treatment with 20 µg NK-Exo for 24 h decreased the number of viable U87MG/F and U87/MG cells by 80%; this result was consistent with the BLI results (Figures S2A,B in Supplementary Material). The MTT assay showed similar results (Figures S2C,D in Supplementary Material). The results of BLI, CCK-8, and MTT analyses confirmed that NK-Exo exerted cytotoxic effects against glioblastoma cells *in vitro*.

**Figure 2:** Natural killer (NK)-Exo cytotoxicity against glioblastoma cells. U87/MG/F cells were cultured with different NK-Exo concentrations, and BLI signals were measured at different time points: **(A)** 6 h, **(B)** 12 h, and **(C)** 24 h. Bio luminescence intensity was quantified using an *in vivo* imaging system and live-imaging software. Experiments were performed in triplicate, and mean ± SD values are plotted. *p < 0.05; **p < 0.01; ***p < 0.001.

RETRACTED

### NK-Exo Uptake by Tumor Cells

To investigate NK-Exo internalization, U87/MG/F cells were treated with DiD-labeled NK-Exo for 1 and 3 h. Confocal laser microscopy detected labeled NK-Exo in cancer cells as early as 1 h after incubation, and the number of exosomes in the cytoplasm of tumor cells increased in a time-dependent manner (Figure 3).

**Figure 3:** Interaction of natural killer (NK)-Exo with glioblastoma cells. U87MGT cells were incubated with phosphate-buffered saline or DiD-labeled NK-Exo (20 μg) for 1 and 3 h, and images were obtained using a confocal laser microscope. Scale bar = 10 μm.

### Effects of NK-Exo on U87/MG/F-Cell Apoptosis

Flow cytometry results showed that NK-Exo induced U87/MG/F-cell apoptosis. U87/MG/F cells were incubated with NK-Exo for 24 h, and annexin V- and PI-labeled cells were counted. Results of annexin V/PI double staining showed increased percentage of necrotic (*p* < 0.05) and apoptotic (*p* < 0.01) cells after NK-Exo treatment. Additionally, NK-Exo treatment decreased the number of living tumor cells compared to the control cells (*p* < 0.001; Figure 4).

**Figure 4:** Natural killer (NK)-Exo induces the apoptosis of glioblastoma cells *in vitro*. **(A)** NK-Exo-induced apoptosis was determined by flow cytometry. **(B)** Quantitative effects are shown in the graph. Apoptosis and necrosis rates in NK-Exo-treated U87/MG/F cells were significantly higher than those in control cells. *p < 0.05; ***p < 0.0001.

To determine the mechanism underlying NK-Exo-induced cancer-cell death, we performed western blot analysis to assess the levels of apoptosis- and cell-proliferation-related proteins (Figures 5A and 6A represent the levels of apoptosis- and cell-proliferation-related proteins, respectively). Glioblastoma cells were incubated with NK-Exo for 24 h, and the levels of caspase-3, cleaved caspase-3, and cleaved PARP were estimated by western blotting. The results showed that cleaved caspase-3 levels were increased by 4.9-fold and cleaved PARP levels were increased by >10-fold in NK-Exo-treated tumor cells compared to that in untreated control cells (Figure 5B). Moreover, western blot analysis showed that p-AKT levels decreased by 62% and p-ERK levels decreased by 44% in NK-Exo-treated tumor cells compared to that in untreated control cells (Figure 6B). However, p38 and PTEN levels increased 1.7- and 37-fold, respectively (Figures 5B and 6B), in NK-Exo-treated tumor cells relative to the control. These results indicate that NK-Exo promoted apoptosis and decreased the proliferation of glioblastoma cells.

**Figure 5:** Effect of natural killer (NK)-Exo on the apoptosis pathway. **(A)** Western blot analysis of marker proteins associated with the apoptosis–signaling pathway. **(B)** Incubation of U87MG/F cells with NK-Exo for 24 h increased the levels of p38, cleaved caspase-3, and cleaved polyADP ribose polymerase.

RETRACTED

**Figure 6:** Effect of natural killer (NK)-Eso on cell proliferation. **(A)** Western blot analysis of marker proteins associated with cell proliferation. **(B)** Incubation of U87MG/F cells with NK-Exo for 24 h decreased p-AKT and p-ERK levels and increased PTETs levels.

### Cytokine and Protein Quantification in NK-Exo

We previously showed that NK-Exo contain the functional proteins FasL and perforin (22); however, the involvement of granzymes in perforin function has not been evaluated (4, 5, 39, 40). We performed an ELISA to confirm the presence of granzyme B in NK-Exo, with the results confirming the presence of granzyme B in NK cells, NK-cell medium, and NK-Exo. In addition, granzyme B levels were higher in NK-Exo than in NK cells (*p* < 0.01) and NK-cell medium (*p* < 0.001) (Figure 7A). Moreover, we detected TNF-α, which is also present in NK cells and induces cytotoxic effects, in NK-Exo (Figure 7B); we also detected perforin and FasL in NK-Exo (Figure 7C), which is consistent with the previous results (22).

**Figure 7:** Cytokines and proteins in natural killer (NK)-Exo. Levels of granzyme B **(A)** and tumor necrosis factor-α **(B)** in NK cells, NK-cell medium, and NK-Exo were measured by enzyme-linked immunosorbent assay. **(C)** Levels of perforin and Fas ligand in NK cells and NK-Exo were measured by western blotting. Experiments were performed in triplicate, and mean ± SD values are plotted. *p < 0.05; **p < 0.001; ***p < 0.0001.

### Biodistribution and *In Vivo* Specificity of NK-Exo Toward Glioblastoma

Both untreated mice and mice pretreated intraperitoneally with dextran sulfate (*n* = 7) were injected with DiD-labeled NK-Exo through the tail vein after 2 h, followed by FLI of NK-Exo both *in vivo* and *ex vivo* after NK-Exo injection (Figure S3 in Supplementary Material). The results of *in vivo* analysis revealed that FLI signals were associated with NK-Exo mainly in the liver and spleen in both groups (with or without dextran sulfate). In addition, NK-Exo showed tumor-specific accumulation as early as 24 h postinjection, and FLI signals in the tumor persisted for >5 days (Figure 8A). Pretreatment with dextran sulfate significantly decreased NK-Exo uptake by the liver and spleen (*p* < 0.0001 and *p* < 0.05, respectively; Figures 8B,C) and increased their uptake by tumor tissue twofold relative to control mice not pretreated with dextran sulfate. Moreover, pretreatment with dextran sulfate prolonged NK-Exo retention in the tumor tissue (Figures 8A,C).

RETRACTED

**Figure 8:** Visualization and *in vivo* tracking of natural killer (NK)-Exo. **(A)** Mice with glioblastoma xenografts (*n* = 7) were injected with DiD-labeled NK-Exo (100 μg) through their tail vein at 2 h after injecting phosphate-buffered saline or dextran sulfate intraperitoneally. **(B,C)** Organs and tumors of the mice were harvested, and fluorescence signals were visualized and quantified using an *in vivo* imaging system. All data are expressed as the mean ± SD from at least three representative experiments. *p < 0.05; **p < 0.01; ***p < 0.001.

Because the BBB inhibits 98% of all methods potentially capable of improving the treatment efficacy in various central nervous system diseases (41–43), we investigated the ability of NK-Exo to cross the BBB. An orthotopic tumor model was successfully established, followed by injection of NK-Exo through the tail vein. Whole-mouse imaging showed a strong fluorescence signal, indicating NK-Exo accumulation in the liver and head areas. To confirm that the signals originated from brain tissue, *ex vivo* brain imaging was performed, revealing that brain tissue showed strong fluorescence both in the presence and absence of a tumor (Figure S4 in Supplementary Material).

### Inhibition of *In Vivo* Tumor Growth by NK-Exo

A schematic diagram of the *in vivo* experiments is shown in Figure 9. Ten days after tumor challenge, mice were randomly divided into three groups (*n* = 6) and injected with 100 μg/150 μL NK-Exo or 150 µL PBS through the tail vein. Furthermore, mice were pretreated with dextran sulfate to inhibit the liver uptake of NK-Exo and enhance the therapeutic effect. BLI performed after seven NK-Exo injections showed significantly lower signals in NK-Exo-injected mice than in PBS-injected mice (*p* < 0.001; Figures 10A,B). Moreover, pretreatment with dextran sulfate increased the immunotherapeutic effect of NK-Exo by inhibiting their liver uptake when compared to NK-Exo treatment alone (*p* < 0.01). In addition, tumor regrowth was observed 1 week after the final NK-Exo injection in mice treated with NK-Exo alone. In contrast, no tumor regrowth was observed, even at 2 weeks postinjection, in mice treated with NK-Exo + dextran sulfate (Figures 10A,B). These results were consistent with those of biodistribution analysis, which showed NK-Exo retention in the tumor tissue for nearly 1 week; however, NK-Exo retention decreased after 5 days in mice treated with NK-Exo alone (Figure 8A).

**Figure 9:** Scheme of *in vivo* experiments to assess the antitumor effect of natural killer (NK)-Exo. To confirm the *in vivo* therapeutic effect of the NK-Exo to the glioblastoma, the xenograft mice was established and randomly divided into three groups (*n* = 6). Phosphate-buffered saline, NK-Exo (100 μg), or NK-Exo combined with dextran was given to each group via intravenous route, respectively. The body weight and the BLI were measured up to 2 weeks after treatment, and at last, *ex vivo* tumor weight was also obtained.

RETRACTED

**Figure 10:** Effects of *in vivo* natural killer (NK)-Exo treatment in the presence and absence of dextran sulfate pretreatment. **(A)** Bioluminescence imaging (BLI) was performed using U87MG/F-cell-injected mice in the control and treatment groups (*n* = 6). Mice in the treatment group were injected with 100 μg NK-Exo through the tail vein every 2 days for 2 weeks. **(B)** Quantification of BLI results. All data are expressed as the mean ± SD from at least three representative experiments. ***p < 0.001 as compared with control mice; ^#^*p* < 0.05, ^##^*p* < 0.01, and ^###^*p* < 0.001 as compared with dextran sulfate-injected mice.

Previous studies have shown that ultrasound imaging provides reliable tumor-volume estimates in animals (44, 45). Therefore, we performed ultrasound imaging after BLI to confirm our results. B-Mode images of the tumor were obtained using an ultrasound imaging system, and a three-dimensional morphology of the tumor was generated. The results of quantitative analysis showed that the volumes of tumors isolated from NK-Exo-alone-treated mice were twofold lower than those of tumors isolated from control mice (26.67 ± 3.16 vs. 57.31 ± 2.15 mm^3^; *p* < 0.001; Figures 11A,B). Moreover, higher antitumor effects were observed in mice treated with NK-Exo + dextran sulfate than in mice treated with NK-Exo alone (6.60 ± 4.23 vs. 26.67 ± 3.16 mm^3^; *p* < 0.01; Figure 11B), which is consistent with the BLI results.

**Figure 11:** *In vivo* ultrasound imaging of tumor and mouse body weight. **(A)** Ultrasound images were obtained in the B mode, and 3D imaging was performed. **(B)** Tumor volumes were measured using software. **(C)** Body weights of mice in each group (*n* = 6) were measured every 4 days until the mice were sacrificed. All data are expressed as the mean ± SD from at least three representative experiments. *p < 0.05; **p < 0.01; ***p < 0.001.

*Ex vivo* BLI was also obtained (Figures 12A,B) and demonstrated that compared with the control group the NK-Exo treatment group showed lower BLI signal. *Ex vivo* tumor weights were consistent with the results of ultrasound imaging (Figure 12C). Tumor weights for control mice were greater than twofold higher than those of mice treated with NK-Exo alone, and mice in the NK-Exo + dextran sulfate group had the smallest tumors. These results supported the results of *in vivo* BLI and ultrasound imaging and indicated the immunotherapeutic efficacy of NK-Exo. Moreover, these results indicated that treatment with an SR-A blocker inhibited liver uptake of NK-Exo and increased their therapeutic effect.

RETRACTED

**Figure 12:** *Ex vivo* tumor measurement. **(A)** Mice (*n* = l 8) were sacrificed, their tumors harvested, and *ex vivo* bioluminescence imaging (BLI) was performed. **(B)** Quantized graph of BLI showing *ex vivo* tumor activity. **(C)** Tumors were weighed using electronic scales. All data are expressed as the mean ± SD from at least three representative experiments, and mean ± SD values are plotted. *p < 0.05; ***p < 0.001.

### Side Effects Associated With NK-Exo

To confirm the safety of NK-Exo, we measured the body weights of mice and performed histological analysis of their vital organs. The body weights of mice treated with NK-Exo alone and NK-Exo + dextran sulfate remained unchanged, suggesting that NK-Exo did not exert any significant cytotoxic effects in mice; however, the body weight of control mice decreased with increasing tumor growth (Figure 11C). Histological analyses of the liver, spleen, lung, and heart tissue isolated from mice treated with NK-Exo alone, and NK-Exo + dextran sulfate were compared to those isolated from healthy mice, at 20× (Figure 13) and 40× magnifications (Figure S5 in Supplementary Material). The results of histological analyses revealed no visible injuries in the liver, lung, spleen, and heart of mice treated with NK-Exo.

**Figure 13:** Histology of vital organs from mice intravenously injected with natural killer (NK)-Exo. To determine the effects of systemic administration of NK-Exo on the vital organs of mice (*n* = 18), the liver, lung, spleen, and heart of NK-Exo-treated mice were harvested on day 29, embedded in paraffin, sectioned, and histologically analyzed. Healthy mice (*n* = 3) not treated with NK-Exo were used as controls.

## Discussion

In this study, we investigated the therapeutic effect of NK-Exo on a glioblastoma cell line using a reporter-gene system by performing CCK-8 and MTT assays *in vitro* and by subjecting the cells to BLI and *in vivo* ultrasound imaging. The mechanism underlying the antitumor effect of NK-Exo was determined by FACS and western blotting, the results of which indicated that NK-Exo induced tumor-cell apoptosis. Furthermore, ELISA detected cytokines present in NK-Exo and aided in the determination of their tumoricidal ability. Moreover, we determined the NK-Exo biodistribution following intravenous administration and their specificity toward glioblastoma in a xenograft mouse model by FLI.

RETRACTED

Natural killer cells function as lymphocytes of the innate immune system and lyse infected cells and tumor cells without sensitization (40, 46, 47). A previous study demonstrated that NK cell therapy is a less toxic alternative to chemotherapy and radiotherapy (48). However, application of primary NK cell-based immunotherapy is limited in treating cancer because of patient variability in cell number and function, inhibition of cytotoxicity by tumors or the tumor microenvironment, and challenges in obtaining sufficient numbers of cells (49). The alternative is to obtain cells from a healthy donor, which requires depletion of allogeneic T cells to prevent graft-versus-host reactions (50). A potential option for overcoming these limitations is the use of a permanent NK cell line. In the current study, we used the human NK cell line NK-92MI. NK-92 is the only malignant permanent NK cell line that has been investigated in clinical trials and confirmed to be safe with no severe side effects (51–53). However, NK-92 cells are highly dependent on cytokine interleukin-2, which exhibits toxicity and may cause capillary leak syndrome (54). NK-92MI cells are not dependent on interleukin-2 and were shown to have an antitumor effect on glioblastoma *in vivo* (6), making them more suitable for this study.

Human NK cells are classified based on their surface expres-sion of CD56 (neural cell adhesion molecule) and lack of CD3 (T-cell co-receptor), and can be categorized into two developmentally related, but functionally distinct, subsets based on relative CD56 expression: CD56^bright^ and CD56^dim^ (55). NK-92 is characterized by the expression of CD56^bright^ and a low level of immunoglobulin G fragment crystallizable region (Fc) receptor (FcγRIII)-CD16, which is typical for a minor subset of NK cells in the peripheral blood (56). However, the CD56^dim^ subset, which expresses maturity-related inhibitory receptors and high surface levels of CD16, as well as permits responses to antibody-opsonized targets, comprises 80–95% of peripheral blood NK cells (57). Moreover, CD56^dim^ NK cells have a higher capacity to recognize and kill target cells, whereas CD56^bright^ NK cells show lower cytotoxicity toward cancer cells because they lack CD16 expression, indicating antibody-dependent cytotoxicity (57). Moreover, NK-92 cells lost the production of interferon-γ, an important activator of macrophages and inducer of major histocompatibility complex class II (58). However, except for these two mechanisms, NK-92 cells could biosynthesize and release granzyme B by secretory lysosomes according to Wang et al. (59), which is consistent with the results of our previous study. Additionally, perforin was detected in NK-92 MI cells and their exosomes. Both granzyme B and perforin showed cytotoxicity toward tumor cells (31, 40, 60). The CD56^bright^ subset possesses distinct chemokine and homing receptor repertoires and produces other cytokines such as TNF-α and granulocyte macrophage colony-stimulating factor unlike CD56^dim^ NK cells (40, 50). These factors may partly explain the tumoricidal ability of NK-Exo; however, detailed studies of the mechanisms are needed to determine function of exosomes derived from NK cells.

RETRACTED

In addition, given the differences in primary NK and NK-92MI cells, exosomes derived from these two cells should be compared. They may also have tumor activity; for example, some tumors express self-HLA, which binds to inhibitory killer immunoglobulin-like receptors to modify the primary NK cells (48). They may also affect the exosomes derived from these cells and, therefore, primary NK cells from the patient should be studied. In conclusion, the biofunction and potency of exosomes derived from primary NK cells of both healthy donors and patients should be explored in the future.

Exosomes are nanovesicles released by cells *in vitro* into the culture medium and *in vivo* into the blood, urine, breast milk, saliva, and malignant effusions (14, 17, 20, 33, 61). Exosomes deliver several molecules, including cytokines, protein, and lipids, to target cells (14, 22, 30, 62) and are approximately 100 nm in size, allowing their interaction with target and barrier cells (9, 25), particularly in the brain (8). Therefore, NK-Exo may represent suitable tools for glioblastoma immunotherapy. Here, NK-Exo were isolated from NK-cell medium by ultracentrifugation and purified by density gradient centrifugation. NK-Exo morphology was determined by TEM (Figure 1A), and NK-Exo size and purity were measured by NTA and DLS as well as western blot analyses, respectively. NTA and DLS results indicated that NK-Exo ranged from 100 to 150 nm in size, and western blot analysis showed that NK-Exo expressed CD63 and Alix (Figure 1), which are exosome marker proteins (9, 18, 24, 61). The nano-size of exosomes allows them to act as passive therapeutic agents for treating various brain diseases (8, 10, 11). Although exosomes have been extensively evaluated, this is the first study assessing their utility for treating glioblastoma.

The antitumor activity of NK-Exo was determined by BLI and cell-proliferation assays (CCK-8 and MTT assays), which showed that treatment with NK-Exo for 24 h decreased the number of tumor cells by 80% (Figure S2 in Supplementary Material). This result is consistent with the FACS results, which showed that NK-Exo treatment decreased the number of living cancer cells by ~50% and increased apoptosis by greater than 13-fold (Figure 4). The current standard NK cytotoxicity estimation method involves a 4-h assay with K562 as a target, enabling the calculation of 51Cr, which should be explored in future studies of NK-Exo. The tumoricidal effect of NK cells involves two major mechanisms: activation of the intrinsic apoptosis pathway, which is induced by perforin and granzymes *via* increased apoptosome formation and caspase-3 activation, and extrinsic apoptosis pathway, which involves caspase-8 and caspase-3 activation (6, 39, 60, 63) (Figure 5A). To explore the mechanism underlying NK-Exo-induced cytotoxicity against tumor cells, we performed ELISA and western blotting, which showed that NK-Exo treatment increased the levels of cleaved caspase-3 and cleaved PARP (Figure 5B) and indicated that NK-Exo induced apoptosis-signaling pathways in tumor cells and initiated cell death. Our previous study showed that NK-Exo contain FasL and perforin (22). In the present study, the ELISA results confirmed the presence of granzyme B and TNF-α in NK-Exo (Figure 7), suggesting their ability to induce the intrinsic apoptosis pathway (31, 32, 60).

RETRACTED

Western blot results indicated that NK-Exo inhibited glioblastoma-cell proliferation by decreasing the levels of p-AKT and p-ERK (Figure 6B), which is consistent with the results of our previous study (22). Another study reported that MSC-derived exosomes inhibit the growth of Lewis lung carcinoma by reducing p-ERK levels (24). The tumor suppressor PTEN is negatively associated with the PI3K/AKT pathway and disrupts cell proliferation by reducing p-AKT levels (35, 36). Moreover, p38 involved in the MAP kinase pathway participates in apoptosis by increasing cleaved caspase-3 levels (64–66). The results of the present study showed that NK-Exo treatment decreased p-AKT (60%) and p-ERK (40%) levels and increased PTEN levels (37%), which inhibited the proliferation and induced the apoptosis of glioblastoma cells. Moreover, NK-Exo treatment increased p38 levels by 1.7-fold, which is consistent with the elevated levels of cleaved caspase-3 and cleaved PARP. These results suggest that NK-Exo induced glioblastoma-cell apoptosis, and that the mechanism underlying the antitumor effect of NK-Exo is related to both increased apoptosis and decreased proliferation of tumor cells. Although the ability of NK-Exo to kill cancer cells and related mechanisms were explored, further studies are needed to confirm the cytotoxic effects of NK-Exo on primary tumors.

The therapeutic effect of NK-Exo against glioblastoma can be improved by understanding the associated *in vivo* kinetics. We previously found that breast cancer-cell-derived exosomes are predominantly distributed in the lungs, a frequent site of metastasis, and directly suppress T cell proliferation and inhibit NK-cell cytotoxicity (67). However, Wiklander et al. (68) showed that the *in vivo* biodistribution of exosomes is associated with the parent cell source, administration routes, and specificity. For example, unlike breast cancer-cell-derived exosomes, which are mainly distributed in the lungs, dendritic cell-derived exosomes typically accumulate in the liver (68). Although immu-notherapy using exosomes has been extensively evaluated (10, 27, 31, 32), the number of studies tracking the *in vivo* distribution of exosomes (24, 69), particularly that of immune-cell-derived exosomes (22, 31, 32), is very limited. However, the hypothesis that immune-cell-derived exosomes can be used for targeting and treating cancers is gaining attention. This is the first study to report the biodistribution of NK-Exo, which can be used as a basis for developing NK-Exo-based treatment strategies.

RETRACTED

The mononuclear phagocyte system plays a major role in clearing systemically delivered exosomes, thereby introducing major barriers to exosome-based therapy (68, 70). Tissue macrophages in the liver and spleen are major components of this system (71), and the results of our study showing accumulation of DiD-labeled NK-Exo in the liver and spleen revealed that NK-Exo are mainly cleared by the mononuclear phagocyte system (Figure 8). A previous study found that the use of dextran sulfate, which inhibits SR-A-family proteins, dramatically decreases the liver uptake and increases the circulation time of exosomes to enhance their accumulation at target sites *in vivo* (21). In the present study, we assessed the spatial and temporal distribution of NK-Exo in both untreated and dextran sulfate pretreated-cells by FLI. In contrast to previous results the exosome started to decrease after 48h, we found the NK-Exo could be detected in the liver, lung and spleen even after 7 days (Figure 8). However, NK-Exo accumulated in the tumor tissue at 24 h; this accumulation is consistent with the results of Watson et al. (21). The results of FLI analysis performed in the present study to determine the biodistribution of DiD-labeled NK-Exo showed the same trend. Intravenous administration of NK-Exo is an ideal route for cancer treatment, as it is feasible in patients with multiple or disseminated metastases or with metastatic lesions at sites where direct injection cannot be performed (67, 72). Therefore, various therapeutic agents are commonly intravenously injected under different clinical conditions. However, the therapeutic effect of new therapeutic agents in preclinical animal studies is verified by their intratumoral injection (24, 68, 73).

RETRACTED

Aggressive treatment can result in serious damage to various organs, such as the liver, heart, lung, intestine, skin, and hematopoietic system, limiting the maximal permissible intensity of treatment and possibly resulting in poor overall survival (74). NK-cell-based treatment is currently being used to treat various incurable malignancies; however, it is associated with significant side effects (54). In the present study, NK-Exo cytotoxicity in mice was determined by measuring their body weight every 4 days until the mice were sacrificed. NK-Exo-treated mice did not show a significant loss of body weight relative to control mice, which showed cachexia because of tumor growth (Figure 11C). Moreover, histological analysis of the vital organs of NK-Exo-treated mice showed that NK-Exo treatment did not exert significant pathological effects (Figure 13; Figure S5 in Supplementary Material). Currently, immunotherapy with NK cells is performed using autologous and allogeneic methods. For autologous treatment, NK cells are expanded *ex vivo* to achieve clinically relevant numbers because of the low number of NK cells in the peripheral or cord blood (60). In contrast, a limited number of NK cells are available for allogeneic treatment because of the lack of donors and requirements for blood-type matching, preventing widespread use of allogeneic NK-cell therapy in oncology clinics (49, 50, 54). Recently, Jong et al. (18) developed a relatively simple and cost-effective method for isolating exosomes from human NK cells on a large scale (18). Moreover, exosome therapy is more advantageous than cell therapy because of the small size of exosomes, which allows them to cross various physiological barriers that cannot be crossed by cells (10, 11, 32, 61, 75, 76). These advantages support the use of NK-Exo as a promising therapeutic tool for treating cancer.

In addition to the innate tumoricidal activity of NK-Exo, exosome therapy can be potentiated through combinatorial use with other therapeutic options. For example, modification of milk-derived exosomes with paclitaxel may increase the aqueous solubility of paclitaxel, efficacy of drug delivery, and efficiency of crossing biological barriers. Moreover, some exosomes can cross the BBB (e.g., macrophage-derived exosomes) and have been successfully used to treat neurodegenerative disorders (11, 17, 69). Exosomes can be loaded with cytokines and miRNAs in addition to chemotherapeutic drugs (27). Dendritic cell- or ascite-derived exosomes loaded with granulocyte/macrophage-colony stimulating factor can be used to treat breast and colorectal cancer, and MSC-derived exosomes loaded with miR-133b, miR-146b, and miR-9 can be used to treat various cancers (10, 16, 25, 77).

RETRACTED

The current clinical applications of exosome research can be categorized into three categories: (1) exosomes as therapeutic agents, (2) exosome-based immunotherapy, and (3) exosome-mediated delivery. Moreover, based on the data in the clinical trials database at the National Institute of Health (http://clinicaltrials.gov), there are several ongoing exosome-based clinical trials that are anticipated to improve survival outcomes for oncological diseases in the near future (62, 76–78). Currently, classic chemotherapeutic drugs function by inducing DNA damage either directly or indirectly. However, tumor cells disrupt their cell cycle checkpoints during tumorigenesis and cannot arrest the cell cycle for a prolonged period, making them resistant to chemotherapy. In addition, prolonged or highly aggressive treatment often results in damage to normal cells in the intestine, skin, and hematopoietic system (74, 79). A previous study suggested that exosomes secreted from monocytes and macrophages can be used to avoid entrapment in mononuclear phagocytes, thereby enhancing the delivery of incorporated drugs to target cells. To this end, a previous study reported the development of a new exosome-based drug-delivery system for treating Parkinson’s disease (11).

Natural killer (NK)-Exo showed strong antitumor activity toward glioblastoma cells both *in vitro* and *in vivo*. Moreover, these exosomes can be loaded with other anticancer agents capable of enhancing their antitumor effect and tumor specificity, or to promote their passage through the BBB. However, additional studies should be performed to confirm and enhance the therapeutic efficiency of NK-Exo for treating incurable glioblastoma and promote the application of NK-Exo therapy in clinical settings.

## Conclusion

Natural killer (NK)-Exo exerted innate therapeutic effects on glio-blastoma both *in vitro* and *in vivo* and dextran sulfate pretreatment enhanced the *in vivo* therapeutic effect of intravenously injected NK-Exo. The *in vivo* kinetics of intravenously injected NK-Exo in the mouse model were successfully monitored by fluorescence imaging, which confirmed the specificity of NK-Exo toward glioblastoma. Moreover, the tumor specificity of NK-Exo was enhanced by blocking SR-A through dextran sulfate pretreatment. Therefore, our results suggest that NK-Exo is a new and promising therapeutic agent for treating incurable glioblastoma.

## Ethics Statement

All animal experiment protocols were conducted in accordance with National Institutes of Health guidelines for the care and use of laboratory animals and approved by the Committee for use Handing and Use of Animals of Kyungpook National University.

RETRACTED

## Author Contributions

LZ: conception and design, execution of experiments, acquisition of data, analysis and interpretation of data, drafting of the manuscript. JO: execution of experiments. PG: analysis and interpretation of data. SK: analysis and interpretation of data. SB: execution of experiments. SJ, S-WL, and JL: critical revision of the manuscript, final approval of the version to be published. B-CA: conception and design, drafting of the manuscript, critical revision of the manuscript, obtained funding, study supervision, final approval of the version to be published, agreement to be accountable for all aspects of the work.

## Conflict of Interest Statement

The authors declare that the research was conducted in the absence of any commercial or financial relationships that could be construed as a potential conflict of interest.

## References

[1] Dunn-PirioAMVlahovicG Immunotherapy approaches in the treatment of malignant brain tumors. Cancer (2016) 123(5):734–50.10.1002/cncr.3037127875627

[2] LeeSJKangWYYoonYJinJYSongHJHerJH Natural killer (NK) cells inhibit systemic metastasis of glioblastoma cells and have therapeutic effects against glioblastomas in the brain. BMC Cancer (2015) 15:1011.10.1186/s12885-015-2034-y26704632PMC4690248

[3] TodaM. Glioma stem cells and immunotherapy for the treatment of malignant gliomas. ISRN Oncol (2013) 2013:673793.10.1155/2013/67379323762610PMC3671309

[4] HwangMHLiXJKimJEJeongSYLeeSWLeeJ Potential therapeutic effect of natural killer cells on doxorubicin-resistant breast cancer cells in vitro. PLoS One (2015) 10(8):e0136209.10.1371/journal.pone.013620926295571PMC4546633

[5] KimHWKimJEHwangMHJeonYHLeeSWLeeJ Enhancement of natural killer cell cytotoxicity by sodium/iodide symporter gene-mediated radioiodine pretreatment in breast cancer cells. PLoS One (2013) 8(8):e70194.10.1371/journal.pone.007019423940545PMC3734030

[6] LeeHWSinghTDLeeSWHaJHRehemtullaAAhnBC Evaluation of therapeutic effects of natural killer (NK) cell-based immunotherapy in mice using in vivo apoptosis bioimaging with a caspase-3 sensor. FASEB J (2014) 28(7):2932–41.10.1096/fj.13-24301424736413

[7] WennerbergEPfefferleAEkbladLYoshimotoYKremerVKaminskyyVO Human anaplastic thyroid carcinoma cells are sensitive to NK cell-mediated lysis via ULBP2/5/6 and chemoattract NK cells. Clin Cancer Res (2014) 20(22):5733–44.10.1158/1078-0432.CCR-14-029125212604

[8] YuanDZhaoYBanksWABullockKMHaneyMBatrakovaE Macrophage exosomes as natural nanocarriers for protein delivery to inflamed brain. Biomaterials (2017) 142:1–12.10.1016/j.biomaterials.2017.07.01128715655PMC5603188

RETRACTED

[9] ChenCCLiuLMaFWongCWGuoXEChackoJV Elucidation of exosome migration across the blood-brain barrier model in vitro. Cell Mol Bioeng (2016) 9(4):509–29.10.1007/s12195-016-0458-328392840PMC5382965

[10] XinHLiYBullerBKatakowskiMZhangYWangX Exosome-mediated transfer of miR-133b from multipotent mesenchymal stromal cells to neural cells contributes to neurite outgrowth. Stem Cells (2012) 30(7):1556–64.10.1002/stem.112922605481PMC3495063

[11] HaneyMJKlyachkoNLZhaoYGuptaRPlotnikovaEGHeZ Exosomes as drug delivery vehicles for Parkinson’s disease therapy. J Control Release (2015) 207:18–30.10.1016/j.jconrel.2015.03.03325836593PMC4430381

[12] LiuYGuYCaoX. The exosomes in tumor immunity. Oncoimmunology (2015) 4(9):e1027472.10.1080/2162402X.2015.102747226405598PMC4570093

[13] GangadaranPHongCMAhnBC. Current perspectives on in vivo noninvasive tracking of extracellular vesicles with molecular imaging. Biomed Res Int (2017) 2017:9158319.10.1155/2017/915831928246609PMC5303595

[14] DaneshAInglisHCJackmanRPWuSDengXMuenchMO Exosomes from red blood cell units bind to monocytes and induce proinflammatory cytokines, boosting T-cell responses in vitro. Blood (2014) 123(5):687–96.10.1182/blood-2013-10-53046924335232PMC3907755

[15] HallJPrabhakarSBalajLLaiCPCerioneRABreakefieldXO. Delivery of therapeutic proteins via extracellular vesicles: review and potential treatments for Parkinson’s disease, glioma, and schwannoma. Cell Mol Neurobiol (2016) 36(3):417–27.10.1007/s10571-015-0309-027017608PMC4860146

[16] MunozJLBlissSAGrecoSJRamkissoonSHLigonKLRameshwarP. Delivery of functional anti-miR-9 by mesenchymal stem cell-derived exosomes to glioblastoma multiforme cells conferred chemosensitivity. Mol Ther Nucleic Acids (2013) 2:e126.10.1038/mtna.2013.6024084846PMC4027430

[17] VashishtMRaniPOnteruSKSinghD. Curcumin encapsulated in milk exosomes resists human digestion and possesses enhanced intestinal permeability in vitro. Appl Biochem Biotechnol (2017) 183(3):993–1007.10.1007/s12010-017-2478-428466459

[18] JongAYWuCHLiJSunJFabbriMWayneAS Large-scale isolation and cytotoxicity of extracellular vesicles derived from activated human natural killer cells. J Extracell Vesicles (2017) 6(1):1294368.10.1080/20013078.2017.129436828326171PMC5345580

[19] Sobo-VujanovicAMunichSVujanovicNL. Dendritic-cell exosomes cross-present toll-like receptor-ligands and activate bystander dendritic cells. Cell Immunol (2014) 289(1–2):119–27.10.1016/j.cellimm.2014.03.01624759079PMC4045011

[20] BretzNPRidingerJRuppAKRimbachKKellerSRuppC Body fluid exosomes promote secretion of inflammatory cytokines in monocytic cells via toll-like receptor signaling. J Biol Chem (2013) 288(51):36691–702.10.1074/jbc.M113.51280624225954PMC3868779

RETRACTED

[21] WatsonDCBayikDSrivatsanABergamaschiCValentinANiuG Efficient production and enhanced tumor delivery of engineered extracellular vesicles. Biomaterials (2016) 105:195–205.10.1016/j.biomaterials.2016.07.00327522254PMC7156278

[22] ZhuLKalimuthuSGangadaranPOhJMLeeHWBaekSH Exosomes derived from natural killer cells exert therapeutic effect in melanoma. Theranostics (2017) 7(10):2732–45.10.7150/thno.1875228819459PMC5558565

[23] PlebanekMPAngeloniNLVinokourELiJHenkinAMartinez-MarinD Pre-metastatic cancer exosomes induce immune surveillance by patrolling monocytes at the metastatic niche. Nat Commun (2017) 8(1):1319.10.1038/s41467-017-01433-329105655PMC5673063

[24] KalimuthuSGangadaranPLiXJOhJMLeeHWJeongSY In vivo therapeutic potential of mesenchymal stem cell-derived extracellular vesicles with optical imaging reporter in tumor mice model. Sci Rep (2016) 6:30418.10.1038/srep3041827452924PMC4958922

[25] KatakowskiMBullerBZhengXLuYRogersTOsobamiroO Exosomes from marrow stromal cells expressing miR-146b inhibit glioma growth. Cancer Lett (2013) 335(1):201–4.10.1016/j.canlet.2013.02.01923419525PMC3665755

[26] ChaputNTaiebJSchartzNFlamentCNovaultSAndreF The potential of exosomes in immunotherapy of cancer. Blood Cells Mol Dis (2005) 35(2):111–5.10.1016/j.bcmd.2005.05.00916027014

[27] PittJMAndreFAmigorenaSSoriaJCEggermontAKroemerG Dendritic cell-derived exosomes for cancer therapy. J Clin Invest (2016) 126(4):1224–32.10.1172/JCI8113727035813PMC4811123

[28] LakhalSWoodMJA. Exosome nanotechnology: an emerging paradigm shift in drug delivery exploitation of exosome nanovesicles for systemic in vivo delivery of RNAi heralds new horizons for drug delivery across biological barriers. Bioessays (2011) 33(10):737–41.10.1002/bies.20110007621932222

[29] ZhuangXYXiangXYGrizzleWSunDMZhangSQAxtellRC Treatment of brain inflammatory diseases by delivering exosome encap-sulated anti-inflammatory drugs from the nasal region to the brain. Mol Ther (2011) 19(10):1769–79.10.1038/mt.2011.16421915101PMC3188748

[30] SharmaPSchiapparelliLClineHT. Exosomes function in cell-cell communication during brain circuit development. Curr Opin Neurobiol (2013) 23(6):997–1004.10.1016/j.conb.2013.08.00523998929PMC3830597

[31] FaisS. NK cell-released exosomes: natural nanobullets against tumors. Oncoimmunology (2013) 2(1):e22337.10.4161/onci.2233723482694PMC3583913

[32] LuginiLCecchettiSHuberVLucianiFMacchiaGSpadaroF Immune surveillance properties of human NK cell-derived exosomes. J Immunol (2012) 189(6):2833–42.10.4049/jimmunol.110198822904309

RETRACTED

[33] TheryCAmigorenaSRaposoGClaytonA. Isolation and characterization of exosomes from cell culture supernatants and biological fluids. Curr Protoc Cell Biol (2006) Chapter 3:Unit 3.22.10.1002/0471143030.cb0322s3018228490

[34] LeeJKParkSRJungBKJeonYKLeeYSKimMK Exosomes derived from mesenchymal stem cells suppress angiogenesis by down-regulating VEGF expression in breast cancer cells. PLoS One (2013) 8(12):e84256.10.1371/journal.pone.008425624391924PMC3877259

[35] ChalhoubNBakerSJ PTEN and the PI3-kinase pathway in cancer. Annu Rev Pathol (2009) 4:127–50.10.1146/annurev.pathol.4.110807.09231118767981PMC2710138

[36] DeGraffenriedLAFulcherLFriedrichsWEGrunwaldVRayRBHidalgoM. Reduced PTEN expression in breast cancer cells confers susceptibility to inhibitors of the PI3 kinase/Akt pathway. Ann Oncol (2004) 15(10):1510–6.10.1093/annonc/mdh38815367412

[37] RouxPPBlenisJ. ERK and p38 MAPK-activated protein kinases: a family of protein kinases with diverse biological functions. Microbiol Mol Biol Rev (2004) 68(2):320–44.10.1128/MMBR.68.2.320-344.200415187187PMC419926

[38] RonkinaNKotlyarovADittrich-BreiholzOKrachtMHittiEMilarskiK The mitogen-activated protein kinase (MAPK)-activated protein kinases MK2 and MK3 cooperate in stimulation of tumor necrosis factor biosynthesis and stabilization of p38 MAPK. Mol Cell Biol (2007) 27(1):170–81.10.1128/MCB.01456-0617030606PMC1800641

[39] TrapaniJASmythMJ. Functional significance of the perforin/granzyme cell death pathway. Nat Rev Immunol (2002) 2(10):735–47.10.1038/nri91112360212

[40] ZhuLLiXJKalimuthuSGangadaranPLeeHWOhJM Natural killer cell (NK-92MI)-based therapy for pulmonary metastasis of anaplastic thyroid cancer in a nude mouse model. Front Immunol (2017) 8:816.10.3389/fimmu.2017.0081628785259PMC5519537

[41] KrollRANeuweltEA. Outwitting the blood-brain barrier for therapeutic purposes: osmotic opening and other means. Neurosurgery (1998) 42(5):1083–99; discussion 1099–100.10.1097/00006123-199805000-000829588554

[42] Dogrukol-AkDBanksWATuncelNTuncelM Passage of vasoactive intestinal peptide across the blood-brain barrier. Peptides (2003) 24(3):437–44.10.1016/S0196-9781(03)00059-712732342

[43] PardridgeWM Drug transport across the blood-brain barrier. J Cereb Blood Flow Metab (2012) 32(11):1959–72.10.1038/jcbfm.2012.12622929442PMC3494002

[44] CheungAMBrownASHastieLACucevicVRoyMLacefieldJC Three-dimensional ultrasound biomicroscopy for xenograft growth analysis. Ultrasound Med Biol (2005) 31(6):865–70.10.1016/j.ultrasmedbio.2005.03.00315936502

[45] WirtzfeldLAWuGBygraveMYamasakiYSakaiHMoussaM A new three-dimensional ultrasound microimaging technology for precli-nical studies using a transgenic prostate cancer mouse model. Cancer Res (2005) 65(14):6337–45.10.1158/0008-5472.CAN-05-041416024636

RETRACTED

[46] LeeHWGangadaranPKalimuthuSAhnBC. Advances in molecular imaging strategies for in vivo tracking of immune cells. Biomed Res Int (2016) 2016:1946585.10.1155/2016/194658527725934PMC5048043

[47] VivierETomaselloEBaratinMWalzerTUgoliniS. Functions of natural killer cells. Nat Immunol (2008) 9(5):503–10.10.1038/ni158218425107

[48] WilliamsBALawADRoutyBdenHollanderNGuptaVWangXH A phase I trial of NK-92 cells for refractory hematological malignancies relapsing after autologous hematopoietic cell transplantation shows safety and evidence of efficacy. Oncotarget (2017) 8(51):89256–68.10.18632/oncotarget.1920429179517PMC5687687

[49] GuillereyCHuntingtonNDSmythMJ Targeting natural killer cells in cancer immunotherapy. Nat Immunol (2016) 17(9):1025–36.10.1038/ni.351827540992

[50] KlingemannHBoisselLToneguzzoF. Natural killer cells for immunotherapy – advantages of the NK-92 cell line over blood NK cells. Front Immunol (2016) 7:91.10.3389/fimmu.2016.0009127014270PMC4789404

[51] AraiSMeagherRSwearingenMMyintHRichEMartinsonJ Infusion of the allogeneic cell line NK-92 in patients with advanced renal cell cancer or melanoma: a phase I trial. Cytotherapy (2008) 10(6):625–32.10.1080/1465324080230187218836917

[52] TonnTSchwabeDKlingemannHGBeckerSEsserRKoehlU Treatment of patients with advanced cancer with the natural killer cell line NK-92. Cytotherapy (2013) 15(12):1563–70.10.1016/j.jcyt.2013.06.01724094496

[53] GellerMACooleySJudsonPLGhebreRCarsonLFArgentaPA A phase II study of allogeneic natural killer cell therapy to treat patients with recurrent ovarian and breast cancer. Cytotherapy (2011) 13(1):98–107.10.3109/14653249.2010.51558220849361PMC3760671

[54] ZamaiLPontiCMirandolaPGobbiGPapaSGaleottiL NK cells and cancer. J Immunol (2007) 178(7):4011–6.10.4049/jimmunol.178.7.401117371953

[55] MichelTPoliACuapioABriquemontBIserentantGOllertM Human CD56bright NK cells: an update. J Immunol (2016) 196(7):2923–31.10.4049/jimmunol.150257026994304

[56] SuckGOdendahlMNowakowskaPSeidlCWelsWSKlingemannHG NK-92: an ‘off-the-shelf therapeutic’ for adoptive natural killer cell-based cancer immunotherapy. Cancer Immunol Immunother (2016) 65(4):485–92.10.1007/s00262-015-1761-x26559813PMC11029582

[57] DuboisSConlonKCMullerJRHsu-AlbertJBeltranNBryantBR IL15 infusion of cancer patients expands the subpopulation of cytotoxic CD56bright NK cells and increases NK-cell cytokine release capabilities. Cancer Immunol Res (2017) 5(10):929–38.10.1158/2326-6066.CIR-17-027928842470PMC8177006

[58] MagisterSTsengHCBuiVTKosJJewettA. Regulation of split anergy in natural killer cells by inhibition of cathepsins C and H and cystatin F. Oncotarget (2015) 6(26):22310–27.10.18632/oncotarget.420826247631PMC4673165

RETRACTED

[59] WangLJiangSXiaoLChenLLiAZhengF. [Rapid biosynthesis and release of 35 kD granzyme B by NK92 cells bypassing secretory lysosomes]. Xi Bao Yu Fen Zi Mian Yi Xue Za Zhi (2016) 32(2):205–11.10.13423/j.cnki.cjcmi.00765726927382

[60] Shoae-HassaniAHamidiehAABehfarMMohseniRMortazavi-TabatabaeiSAAsgharzadehS. NK cell-derived exosomes from NK cells previously exposed to neuroblastoma cells augment the antitumor activity of cytokine-activated NK cells. J Immunother (2017) 40(7):265–76.10.1097/CJI.000000000000017928622272PMC7543683

[61] MunagalaRAqilFJeyabalanJGuptaRC. Bovine milk-derived exosomes for drug delivery. Cancer Lett (2016) 371(1):48–61.10.1016/j.canlet.2015.10.02026604130PMC4706492

[62] YuDDWuYShenHYLvMMChenWXZhangXH Exosomes in development, metastasis and drug resistance of breast cancer. Cancer Sci (2015) 106(8):959–64.10.1111/cas.1271526052865PMC4556383

[63] AugsteinPHeinkePSchoberCSalzsiederE. Impact of cytokine- and FasL-induced apoptosis in the beta-cell line NIT-1. Horm Metab Res (2009) 41(3):207–12.10.1055/s-0028-109334318975252

[64] CargnelloMRouxPP. Activation and function of the MAPKs and their substrates, the MAPK-activated protein kinases. Microbiol Mol Biol Rev (2011) 75(1):50–83.10.1128/MMBR.00031-1021372320PMC3063353

[65] HeffronDMandellJW. Differential localization of MAPK-activated protein kinases RSK1 and MSK1 in mouse brain. Brain Res Mol Brain Res (2005) 136(1–2):134–41.10.1016/j.molbrainres.2005.01.01415893597

[66] GaestelM. MAPK-activated protein kinases (MKs): novel insights and challenges. Front Cell Dev Biol (2015) 3:88.10.3389/fcell.2015.0008826779481PMC4705221

[67] WenSWSceneayJLimaLGWongCSBeckerMKrumeichS The biodistribution and immune suppressive effects of breast cancer-derived exosomes. Cancer Res (2016) 76(23):6816–27.10.1158/0008-5472.CAN-16-086827760789

[68] WiklanderOPNordinJZO’LoughlinAGustafssonYCorsoGMagerI Extracellular vesicle in vivo biodistribution is determined by cell source, route of administration and targeting. J Extracell Vesicles (2015) 4:26316.10.3402/jev.v4.2631625899407PMC4405624

[69] AgrawalAKAqilFJeyabalanJSpencerWABeckJGachukiBW Milk-derived exosomes for oral delivery of paclitaxel. Nanomedicine (2017) 13(5):1627–36.10.1016/j.nano.2017.03.00128300659

[70] ImaiTTakahashiYNishikawaMKatoKMorishitaMYamashitaT Macrophage-dependent clearance of systemically administered B16BL6-derived exosomes from the blood circulation in mice. J Extracell Vesicles (2015) 4:26238.10.3402/jev.v4.2623825669322PMC4323410

RETRACTED

[71] Mil’toIV. [Liver, lung, kidney and spleen macrophages in rats after intravenous administration of the modified magnetite nanoparticles]. Morfologiia (2014) 146(5):40–5.25823288

[72] LimSMShinSJChungWYParkCSNamKHKangSW Treatment outcome of patients with anaplastic thyroid cancer: a single center experience. Yonsei Med J (2012) 53(2):352–7.10.3349/ymj.2012.53.2.35222318823PMC3282954

[73] SunDZhuangXXiangXLiuYZhangSLiuC A novel nanoparticle drug delivery system: the anti-inflammatory activity of curcumin is enhanced when encapsulated in exosomes. Mol Ther (2010) 18(9):1606–14.10.1038/mt.2010.10520571541PMC2956928

[74] JangSCKimOYYoonCMChoiDSRohTYParkJ Bioinspired exosome-mimetic nanovesicles for targeted delivery of chemotherapeutics to malignant tumors. ACS Nano (2013) 7(9):7698–710.10.1021/nn402232g24004438

[75] GilliganKEDwyerRM. Engineering exosomes for cancer therapy. Int J Mol Sci (2017) 18(6).10.3390/ijms1806112228538671PMC5485946

[76] Rufino-RamosDAlbuquerquePRCarmonaVPerfeitoRNobreRJde AlmeidaLP. Extracellular vesicles: novel promising delivery systems for therapy of brain diseases. J Control Release (2017) 262:247–58.10.1016/j.jconrel.2017.07.00128687495

[77] EscudierBDorvalTChaputNAndreFCabyMPNovaultS Vaccination of metastatic melanoma patients with autologous dendritic cell (DC) derived-exosomes: results of thefirst phase I clinical trial. J Transl Med (2005) 3(1):10.10.1186/1479-5876-3-1015740633PMC554765

[78] BastosNRuivoCFSilvaSMeloSA. Exosomes in cancer: use them or target them? Semin Cell Dev Biol (2017).10.1016/j.semcdb.2017.08.00928803894

[79] KimOYChoiSJJangSCParkKSKimSRChoiJP Bacterial protoplast-derived nanovesicles as vaccine delivery system against bacterial infection. Nano Lett (2015) 15(1):266–74.10.1021/nl503508h25506626

